# Cardiovascular and Metabolic Diseases Etiology Research Center (CMERC) cohort: study protocol and results of the first 3 years of enrollment

**DOI:** 10.4178/epih.e2017016

**Published:** 2017-04-01

**Authors:** Jee-Seon Shim, Bo Mi Song, Jung Hyun Lee, Seung Won Lee, Ji Hye Park, Dong Phil Choi, Myung Ha Lee, Kyoung Hwa Ha, Dae Jung Kim, Sungha Park, Won-Woo Lee, Hyeon Chang Kim

**Affiliations:** 1 Department of Preventive Medicine, Yonsei University College of Medicine, Seoul, Korea; 2 Cardiovascular and Metabolic Diseases Etiology Research Center, Yonsei University College of Medicine, Seoul, Korea; 3 Department of Public Health, Yonsei University Graduate School, Seoul, Korea; 4 Department of Endocrinology and Metabolism, Ajou University School of Medicine, Suwon, Korea; 5 Cardiovascular and Metabolic Disease Etiology Research Center, Ajou University School of Medicine, Suwon, Korea; 6 Division of Cardiology, Severance Cardiovascular Hospital and Cardiovascular Research Institute, Yonsei University College of Medicine, Seoul, Korea; 7 Department of Microbiology and Immunology, Seoul National University College of Medicine, Seoul, Korea; 8 Department of Biomedical Sciences, Seoul National University College of Medicine, Seoul, Korea

**Keywords:** Cardiovascular diseases, Metabolic diseases, Cohort studies, Korea

## Abstract

Although the etiologies of cardiovascular disease (CVD) are widely understood, the goal of finding a globally effective solution for preventing CVD is unrealistic. Therefore, we aimed to conduct a community-based prospective study on the prevention and management of CVD in Korean adults. This study was designed to recruit 8,000 healthy adults over the course of 5 years. The baseline assessment includes a wide range of established CVD risk factors, including demographic characteristics, medical history, health behaviors, psychological conditions, body size and composition, blood pressure, the augmentation index, carotid ultrasonography, an electrocardiogram, and biochemical indicators, as well as some novel factors, such as social network characteristics, exposure to environmental pollutants, inflammatory markers, hemostatic markers, and immunosenescence markers. Annual telephone interviews and follow-up health examinations at 5-year intervals after the baseline assessment are planned to collect information on changes in health status and its determinants. Additionally, indirect follow-up using secondary data sources will be conducted to obtain information on health services utilization and death. So far, more than 6,000 adults have been enrolled during the first three and a half years, and almost all participants have been tracked by annual telephone follow-up surveys. The data have been uploaded to iCReaT, the clinical research information management system of the Korea National Institute of Health.

## INTRODUCTION

Cardiovascular disease (CVD), including ischemic heart disease and stroke, is the leading cause of death in the world [1]. Over the past three decades in Korea, ischemic heart disease mortality has increased, whereas stroke mortality has markedly decreased but still remains the top cause of death [2,3]. During the same period, the prevalence of obesity and diabetes has consistently increased among Koreans [4]. Fortunately, CVD is preventable with the management of health-related behaviors and the treatment of existing risk factors. Thus, it is important to identify high-risk individuals who merit lifestyle modification and preventive treatment for the primary prevention of CVD, and risk assessment tools have been developed to predict an individual’s CVD risk for a specific period [5,6]. In Korea, the burdens of CVD and metabolic disorders are expected to steadily increase, in correspondence with the rapid aging of the population and lifestyle changes. It is known that the distributions of traditional risk factors, including smoking, diabetes, hypertension, diet, exercise, and alcohol drinking, as well as genetic traits, their impact on disease development, and disease frequencies vary by region, race, culture, and environment [7]. The goal of finding a globally effective solution for disease prevention is therefore unrealistic [8]. Thus, studies are still needed in various settings to find new determinants, including social, biological, and environmental factors.

The Cardiovascular and Metabolic Diseases Etiology Research Center (CMERC) was funded by the Ministry of Health and Welfare of the Korean Government in 2013 to conduct a new cohort study. The ultimate goals of the CMERC study are to identify novel risk factors and biomarkers for CVD, to measure the contribution of known CVD risk factors to the disease, to develop improved CVD prediction tools for the Korean population, and to produce evidence regarding the preventive treatment of CVD. Ultimately, the study findings will improve our ability to identify high-risk individuals who merit earlier intervention, to develop evidence-based preventive strategies, and to reduce the socioeconomic burden of CVD and metabolic diseases. To achieve these goals, the CMERC designed 2 prospective cohorts: a general-population cohort (the CMERC cohort) and a cohort of high-risk patients (the CMERC-HI cohort).

## STUDY PARTICIPANTS

The CMERC cohort was designed to recruit 8,000 community-living individuals free from myocardial infarction, heart failure, or stroke. Enrollment of the cohort participants and data collection are conducted in two research clinics, operated by the Department of Preventive Medicine, Yonsei University College of Medicine (YUCM), Seoul, Korea and the Department of Endocrinology and Metabolism, Ajou University School of Medicine (AUSM), Suwon, Korea. Participants are recruited mainly through advertisements in the regional newspapers, promotional posters in public areas, or through the acquaintances of study participants. The inclusion and exclusion criteria were designed to maximize the recruitment of community-dwelling middle-aged adults, and to minimize the effects of pre-existing diseases and loss to follow-up (Table 1). The CMERC cohort started participant recruitment and baseline examinations in December 2013, and enrollment is expected to be completed in June 2018. So far, more than 6,000 adults have been enrolled during the first 3 and a half years. Table 2 shows the characteristics of the CMERC cohort participants enrolled for the first 3-year and those of the general population in the same age ranges, analyzed using data from the Korea National Health and Nutrition Examination Surveys (KNHANES) 2013-2014. Compared with the characteristics of the general population, the CMERC cohort participants are more likely to be female and older, but are more educated, comprise more white-collar workers, have a higher income, and engage in more healthy lifestyle-related behaviors, reflecting the characteristics of the urban middle class in Korea.

The CMERC-HI cohort, a sister study of the CMERC cohort, was planned to enroll another 4,000 patients who are at a high risk of developing myocardial infarction or stroke. Patient enrollment for the CMERC-HI cohort is conducted by the Division of Cardiology, Severance Cardiovascular Hospital, YUCM, and the study protocol will be reported separately elsewhere.

### Ethical considerations

This study has been approved by the institutional review boards of Severance Hospital, Yonsei University Health System, Seoul, Korea (4-2013-0661) and Ajou University Hospital, Suwon, Korea (AJIRB-BMR-SUR-13-272). Written informed consent has been obtained from all participants prior to the baseline survey. Participants have been informed that they can withdraw from the study at any time.

## MEASUREMENTS

### Screening and baseline assessment

The CMERC cohort was designed to enroll 4,000 community-living adults at each clinic over 5-year, resulting in a total of 8,000 participants. The baseline assessment includes demographic characteristics, medical history, health behaviors, psychological conditions, social network characteristics, anthropometric measures, resting blood pressure (BP), radial pulse tonometry, carotid artery ultrasonography, an electrocardiogram, bone densitometry, body composition, and biochemical analyses of a fasting blood sample and a casual urine specimen. Both research clinics share the same study protocol, meaning that majority of the baseline assessments and laboratory tests have been standardized (Table 3). However, each clinic has additional laboratory and imaging tests for center-specific research purposes (Table 4). For example, the YUCM clinic additionally measures blood troponin and some inflammatory biomarkers, while the AUSM clinic additionally measures blood concentrations of heavy metals and persistent organic pollutants. Prior to the beginning of cohort enrollment, standardized questionnaires and measurement protocols were established. All interviewers and examiners are required to complete a 3-day course of education on the process of interviewing and conducing a medical examination, and to pass a qualifying test after the education. The questionnaire-based interview and health examination are performed on the same day. All participants are required to fast for at least 8-hour before visiting the research clinic, and to wear a designated lightweight gown during the examination process.

#### Demographic characteristics and medical history

Demographic data on sex, age, education, marriage, cohabitation during the past year, occupation, household income, and subjective economic status are collected. The medical history covers the participant’s history of diseases, family history, medication, and female reproductive factors. The presence of a diagnosis by a physician and the age at the first diagnosis of each of the following diseases are investigated: stroke, transient ischemic attacks, myocardial infarction, angina pectoris, heart failure, chronic kidney disease, hypertension, dyslipidemia, diabetes, thyroid disease, fatty liver, chronic hepatitis, liver cirrhosis, asthma or chronic obstructive pulmonary disease, osteoporosis, arthritis, autoimmune disease, and malignant tumors. If a participant reports a history of stroke, myocardial infarction, heart failure, or active cancer, he/she is excluded from the study. Participants are also required to report whether a family member (father, mother, and siblings) has been diagnosed with or died from specific diseases (myocardial infarction, hypertension, stroke, or diabetes), and to provide their family member’s age at the first diagnosis of the disease or at death. Female participants are required to provide additional information on reproductive health, including age at menarche, menstruation during the past 3-month, menopause, age at menopause, number of pregnancies (total, childbirth, miscarriage, and stillbirth), the presence of gestational diabetes or hypertension, oral contraceptive use, and female hormone use.

#### Health behaviors

Information on cigarette smoking and alcohol drinking are collected using standardized questions that gather information about lifetime smoking, current smoking, age at smoking initiation, the amount and duration of smoking, lifetime drinking, current drinking, and frequency of consumption and average amount consumed of each type of alcohol. Dietary exposures are evaluated using a semi-quantitative food frequency questionnaire (FFQ) that was developed and validated for the KNHANES [9]. The FFQ asks for participants’ average consumption frequency and amount of 112 food items during the preceding year [10]. The FFQ has an acceptable level of validity and reliability for assessing usual dietary intake [11]. Physical activity is evaluated using a Korean version of the International Physical Activity Questionnaire-Short Form [12], which asks for the frequency of each activity (walking, moderate-intensity activity, and vigorous activity) and the duration thereof during the past 7-day. The sleep questionnaire covers quantity (bedtime, rise time, sleep duration) and quality (difficulty in falling asleep, and in sleeping again after waking) of sleep and a screening for obstructive sleep apnea known as the Berlin questionnaire [13]. All the health behaviors listed above are obtained based on participants’ subjective reports through a face-to-face interview. Additionally, physical activity and sleep habits are measured using a wrist-worn accelerometer (GENEActive, Activinsight, Kimbolton, Cambridge, UK) for a subsample of the participants at the YUCM clinic. The device applied in this study is a 3-axial seismic acceleration sensor housed in a small (43×40×13 mm), lightweight (16 g), and waterproof case, and makes objective measurements of participants’ free-living physical activities [14]. To assess participants’ usual data on sleep and physical activity, they are required to wear the device for seven consecutive days, and also to record a log of details about how they wore the device, such as the time of detachment/reattachment and the reason for putting it on or taking it off.

#### Psychological condition and cognitive function

Depressive symptoms and psychosocial responses to stress are assessed in a self-administered manner, not by a face-to-face-interview, and all answers are reviewed by research personnel to check for any instances of misreading, miswriting, or missing answers. Depressive symptoms during the past 2-week are assessed using the Korean version [15] of the Beck Depression Inventory-II [16], which contains 21 questions that reflect the physical and psychological aspects of depression. We also collect participants’ general psychosocial response to stress during the past 6-month, using the Korean version of the life experiences survey questionnaire [17]. The original questionnaire lists 57 possible life events, such as marriage, divorce, death of family members or friends, lifestyle changes, and educational and occupational successes and failures [18]. Of the 57 total events, 10 items that are applicable to students have been omitted in this study, and participants are additionally asked to report any important event not included in the list of 47. Participants are asked to report the presence of stressful life events and the positive or negative effects of each life event. Cognitive function is assessed only for participants aged 50 years or older using the Korean version of the Mini-Mental State Estimation for dementia screening [19]. This questionnaire includes psychometric properties such as orientation to time, place, and person; verbal memory; concentration and calculation; and the functions of language, praxis, and visuospatial construction.

#### Social network analysis

We collect information about social network properties and social support via face-to-face interviews. For the measurement of social network properties, we use questionnaires that were developed for the US. General Social Survey [20] and National Social Life, Health, and Aging Project [21], and translated into the Korean language for the Korean Social Life, Health, and Aging Project [22]. Collecting a complete graph of the social network for all people in a specific community can generate all the social relations between all the people in the community. This type of social network is a complete network or a global network. In contrast, collecting network data from a sample of the population produces a more limited number of networks, in which only the respondent and his or her own social network members are listed. This type of social network is an ego-centric network that consists of the respondent (ego) and his or her social network members (alters). The CMERC cohort measures the ego-centric social networks of the participants. Participants are asked to list their spouse, acquaintances (up to 5) with whom they have discussed important matters, and another individual not in the list of up to 5 members provided earlier but still close and important to the participant. The following question is used to identify acquaintances: “*From time to time, most people discuss things that are important to them with others. For example, these may include good or bad things that happen to you, problems you are having, or important concerns you may have. Looking back over the last 12 months, who are the people with whom you most often discussed things that were important to you?*” They are also asked to provide information about their relationship with each network member, each network member’s demographic characteristics, such as sex, age, cohabitation status, and educational status, how often they talk to (or meet) each network member, and the degree to which they feel emotional closeness to each network member. In addition, they are asked for information about social interactions among the members of their social network.

Analyzing the collected information, we can measure ego-centric network properties, consisting of the participant (ego) and his or her social network member (alters) including network size, network density, content, composition, emotional closeness of alters, volume of contact with alters, bridging potential, and many others. More details regarding the data collection procedures and measurement of social network properties were presented in a previous study [22].

#### Anthropometric measurements

Height is measured to the nearest 0.1 cm using stadiometers: a DS-102 (Jenix, Seoul, Korea) and a BSM-330 (Inbody, Seoul, Korea) in the YUCM clinic, and a BSM-330 (Inbody) in the AUSM clinic. Body weight is measured to the nearest 0.1 kg on a digital scale: a DB-150 (CAS, Seongnam, Korea) and a BSM-330 (Inbody) in the YUCM clinic, and a BSM-330 (Inbody) in the AUSM clinic. Although the stadiometers and weight scale are not identical in the two research clinics, the measurement is made according to a standardized protocol. In addition, a zero-point adjustment is conducted in the same manner at least once a week using a standard ruler (170 cm) and weights (20, 40, and 60 kg). Body circumferences are measured to the nearest 0.1 cm using a plastic measuring tape (SECA 201, SECA, Hamburg, Germany), while maintaining the level of the measuring tape. Waist circumference is measured at the midpoint between the lower point of the rib cage and the upper point of the iliac crest during exhalation. Hip circumference is measured at the widest region of the hip. Mid-thigh circumference is measured at the midpoint between the inguinal crease of the right leg and the proximal border of the patella in a standing position with feet 20 cm apart and the right foot in front of the left. Mid-arm circumference is measured at the midpoint of the right arm between the acromion and the olecranon.

#### Blood pressure measurements

Single arm BP is measured in the right arm in both clinics. Participants take at least a 5-minute rest in the seated position and they are asked to remain still and relaxed during all measurements. A cuff tailored to their individual mid-arm circumference is used, and trained research personnel conduct BP measurements using an automated oscillometric device (HEM-7080, Omron Health, Matsusaka, Japan) in accordance with a standardized protocol. Systolic and diastolic blood pressures are measured three times at 2-minute intervals in the right arm. Measurements are made on the left arm only if right arm measurements are impossible. Additionally, at the YUCM clinic, dual-arm BP measurements are made three times at 60-second intervals, using a device with two cuffs developed for simultaneous dual-arm measurements (WatchBP Office, Microlife, Widnau, Switzerland) [23]. At the YUCM clinic, radial arterial pulse waves are measured and the augmentation index is calculated using a non-invasive device (HEM-9000 AI, Omron Health).

#### Carotid artery ultrasonography

Carotid artery ultrasonography is performed at both research clinics, and all operators have been trained according to a predefined study protocol. However, the ultrasonography machines are not identical at the YUCM clinic (Accuvix XG, Samsung Medison, Seoul, Korea) and the AUSM clinic (Logiq S8 ECG module, GE Healthcare, Chalfont St. Giles, UK). While being measured, participants are in the supine position with their neck extended and their head turned 30° toward the opposite direction of the measurement site. Carotid intima-media thickness (CIMT) is scanned at the 1-cm segment of the common carotid arteries proximal to the bulb region, at the time of the R-wave on the electrocardiogram, and is calculated using the dedicated software installed in the equipment in each clinic. The mean and maximum CIMT values are measured on both the right and left sides. A carotid artery plaque is considered present if the thickness is greater by 50% or more than the surrounding intima-media thickness, or if its size is 1.5 mm or more. The presence and thickness of a carotid plaque is observed by an operator and assessed in both the right and left common, external, and internal carotid arteries, as well as at the bulb area. More details and the inter-rater reliability of the CIMT measurements have been reported separately [24].

#### Electrocardiography

Resting electrocardiography is conducted in the supine position using a standard 12-lead electrocardiogram. The electrocardiography machines used in this study are made by the same company, but the model numbers are different in the YUCM clinic (MAC-5500, GE Healthcare, Chicago, IL, USA) and the AUSM clinic (MAC-3500, GE Healthcare).

#### Bone densitometry

Participants’ bone mineral density is measured by quantitative computerized tomography (QCT) at the YUCM clinic, and by whole body dual-energy X-ray absorptiometry (DXA) at the AUSM clinic. At the YUCM clinic, the bone mineral density of the lumbar spine (T12-L2) and hip is measured using a Somatom Definition AS+ 128 channel CT (Siemens Healthcare, Forchheim, Germany), a Somatom sensation 64 channel CT (Siemens Healthcare), or a GE Lightspeed VCT apparatus (General Electric Medical System, Milwaukee, WI, USA). Scanning is done at 120 kV and 150 mAs and images are reconstructed with a 3-mm slice thickness. All scanned data are analyzed using the QCT PRO software (Mindways Software, Austin, TX, USA) and the CTXA Hip Exam Analysis protocol (Mindways Software). The AUSM clinic measures bone mineral density using whole-body DXA scans (Lunar iDXA, GE Healthcare, Madison, WI, USA), and the acquired data are analyzed with the enCORE software (GE Healthcare). A trained operator conducts all examination procedures according to the standardized protocol of each clinic.

#### Body composition

Bioimpedance analysis is used to assess participant’s body composition parameters, such as body fat and muscle content. During the test, participants hold onto hand electrodes and stand barefoot on the foot electrodes, and spread out their arms and legs naturally.

Different models from the same company were used for measuring bioimpedance: the InBody 370 (Biospace Co., Seoul, Korea) at the YUCM clinic and the Inbody 720 (Biospace Co.) at the AUSM clinic. Both machines estimate information about body circumference (chest, waist, hip right arm, left arm, right thigh, and left thigh) and the body composition of each location (right arm, left arm, trunk, right leg, and left leg), as well as estimating total body composition (body fat, fat-free mass, and total body water). These properties are measured across the same wide range of frequencies (5, 50, and 250 kHz). In addition to the bioimpedance analysis, QCT or DXA is also used to measure body composition. The YUCM clinic assesses abdominal adipose tissue distribution, mid-thigh muscle, and liver adiposity using QCT. Images scanned at the lumbar spine, the L1 level, and the L4 level, are used to estimate the amount of visceral and subcutaneous fat and to confirm the presence of fatty liver, respectively. Voxels are separated into fat and muscle tissue by Hounsfield units (HU): −190 to −30 HU for fat and 0 to 100 HU for muscle. The AUSM clinic estimates total mass, tissue mass, lean mass, and fat mass using the DXA android region of interest [25].

#### Biochemical tests

Overnight-fasting blood samples and casual urine samples are obtained in the morning, and bioassays are performed at a single laboratory (Seoul Clinical Laboratories R&D Center, Seoul, Korea). Concentrations of blood glucose, blood urea nitrogen, creatinine, uric acid, total protein, and albumin are evaluated using a colorimetric method with an analyzer (ADIVA 1800 AutoAnalyzer, Siemens Medical Sol., Deerfield, IL, USA). Insulin levels are determined using a radioimmunoassay with a SR-300 apparatus (Stratec, Birkenfeld, Rhineland-Palatinate, Gemany). Lipid profiles, including total cholesterol, triglycerides, high-density lipoprotein cholesterol and low-density lipoprotein cholesterol levels, and liver function indices, including aspartate aminotransferase, alanine aminotransferase, and γ-glutamyl transferase, are analyzed enzymatically with an ADIVA 1800 AutoAnalyzer (Siemens Medical Sol.). The blood concentration of 25-hydroxy vitamin D is assessed by a chemiluminescence immunoassay using a Liason apparatus (Diasorin, Darmstadt, Hesse, Germany). High-sensitivity C-reactive protein is evaluated using the turbidimetry method with an ADIVA 1800 AutoAnalyzer (Siemens Medical Sol.). Hemoglobin A1c is determined using high-performance liquid chromatography with a Variant II Turbo (Bio-Rad, Hercules, CA, USA). Complete blood cell counts are determined using flow cytometry with an ADIVA 2120i (Siemens, Medical Sol.). Routine urinalysis is done using a urine reagent strip test with a Uriscan Pro II apparatus (YD Diagnostics, Yonginsi, Korea). The AUSM clinic additionally performs an oral glucose tolerance test, with measurements of blood glucose and insulin levels 0, 30, 60, and 120 minutes after a 75-g glucose load. The YUCM clinic additionally measures inflammatory and hemostatic markers, including prothrombin time, activated partial thromboplastin time, factor VII, factor VIII, fibrinogen, fibrin D-dimer and high sensitive troponin T in a subset of enrolled participants.

#### Immunosenescence biomarkers

We measure cellular immunity and immunosenescence biomarkers, such as CD4, CD8, CD28, and IL-6. These immunological characteristics and clinical features are analyzed using fluorescence-activated cell sorting analysis and enzyme-linked immunosorbent assays [26] for subsamples of the participants enrolled at each clinic. Chronic inflammation has been established to be responsible for the development of CVD [27], meaning that it may be a therapeutic target.

### Follow-up assessments

Cohort participants will be followed up directly and indirectly. To collect information on changes in health status and its determinants directly, we plan to conduct telephone interviews and follow-up health examinations. Every participant is contacted annually in a phone interview to check for changes in address and phone number, new disease diagnoses, hospitalizations, and deaths. A few weeks prior to the phone call, a letter informing participants about the upcoming call is delivered to the participants’ home address. Trained interviewers conduct the telephone interviews according to a predetermined protocol. So far, the response rate has remained quite high, due to the enthusiastic efforts of the research staff, with response rates of 99.7% for the first follow-up and 99.3% for the second follow-up [28]. Follow-up health examinations are planned to be conducted every 5-year after the baseline assessment. In addition to the direct follow-up surveys described above, indirect follow-up using secondary data sources such as the National Health Insurance claims database, National Death Statistics, and the National Cancer Registry is planned to obtain information on health services utilization and mortality.

## KEY FINDINGS

The cohort enrollment of this study is currently underway, and will be completed in the middle of 2018. The baseline assessments have not ended yet and sufficient follow-up observations have not been made, meaning that it has not yet become possible to carry out studies to identify new risk factors for CVD. Some cross-sectional analyses using the collected baseline data have been conducted and their results have been reported [23-25,29].

## STRENGTHS AND WEAKNESSES

The CMERC cohort collects plentiful information on emerging risk factors and biomarkers, as well as established traditional risk factors of CVD and metabolic diseases. The analysis of individuals’ social networks in the general Korean population is a strong point of this study, since the relationships between social network characteristics and physical health have not been appropriately studied in Korea. While macro-level socioeconomic factors are difficult to modify, social network characteristics can be partially modifiable, and thus can be used directly to prevent disease. Analyses of cellular immunity and immunosenescence biomarkers are another unique feature of this study. Immunosenescence has been studied as a new important mechanism for chronic diseases, and there is a possibility of finding potential therapeutic candidates targeting immunosenescence. The CMERC cohort has limited generalizability, since it is not randomly drawn from the target population. This study focused on enhancing the diversity of exposure levels rather than on the pure representativeness of the sample. Another limitation is the standardization of risk factor measurement. Some measurements have not been not fully standardized, especially those that require expensive equipment, such as imaging studies.

## DATA ACCESSIBILITY

We have uploaded data for each survey year to iCReaT, the clinical research information management system of the Korea National Institute of Health. We also keep biospecimens such as serum, plasma, buffy coat, and urine for future use, after obtaining individual consent for the retention period and scope of use. Biospecimens will be deposited at the Korea Biobank, managed by the Korea Centers for Disease Control and Prevention, after completion of the baseline assessment. Although cohort enrollment and baseline assessment are ongoing, this study is open to interested researchers. Researchers interested in collaborative study are invited to contact the CMERC principal investigator, Hyeon Chang Kim, at hckim@yuhs.ac.

## Figures and Tables

**Table 1.** Eligibility criteria for the cohort participants

	Criteria
Inclusion	Aged 30 to 64 years
	Living in the current place of residence for at least 8 mo/yr
	No plan to move out of the study area within 2 years
	Able to articulate their own opinions regarding study participation
Exclusion	Diagnosed with cancer within 2 years or still undergoing cancer treatment
	History of myocardial infarction, stroke, or heart failure
	Participating in any randomized clinical trials
	Currently pregnant

**Table 2.** General characteristics in the baseline survey of the CMERC cohort participants for the first 3 years and comparison with the general population in Korea

	CMERC cohort (n=4,890)		General population^1^ (n=7,247)	
	Male (n=1,774)	Female (n=3,116)	Male (n=3,077)	Female (n=4,170)
Sex	36.3	63.7	50.5	49.5
Age (yr)	49.3	50.5	46.0	46.2
30-39	22.4	15.4	29.8	28.9
40-49	23.9	24.1	32.1	31.7
50-59	36.0	46.1	29.1	29.6
60-64	17.6	14.4	9.0	9.7
Marital status, married	94.4	96.5	88.4	94.6
Educational status				
≤ Elementary school	2.9	7.0	8.1	13.9
Middle or high school	40.6	57.4	46.2	51.3
≥ College	56.5	35.7	45.8	34.8
Income (10,000 KRW/mo)	586.4	518.3	424.0	411.0
Occupation				
White collar	49.9	25.5	36.7	20.9
Pink or blue collar	42.0	29.9	52.2	33.4
Unemployed	8.1	44.6	11.1	45.8
Current smoker	35.3	3.1	47.6	4.9
Lifetime alcohol drinker	89.9	66.8	92.9	84.3
Obesity^2^	48.9	27.4	41.7	26.1
Hypertension^3^	31.0	19.5	28.7	16.9
Diabetes mellitus^4^	9.2	5.1	11.5	6.3
Hypercholesterolemia^5^	16.1	19.5	13.8	14.0
Hypertriglyceridemia^6^	27.6	17.3	27.6	10.0
Low HDL cholesterol^7^	18.6	6.2	37.4	16.5

Values are presented as % or mean. CMERC, Cardiovascular and Metabolic Diseases Etiology Research Center; HDL, high-density lipoprotein; KRW, Korean won.

1 Source from Korea National Health and Nutrition Examination Survey (KNHANES, 2013-2014). The results in this table showed distributions and means among adults between 30 and 65 years of age.

2 Obesity was defined as a body mass index ≥25.0 kg/m^2^.

3 Hypertension as treatment with medication or a systolic blood pressure reading of ≥140 mmHg or a diastolic blood pressure of ≥90 mmHg.

4 Diabetes mellitus as treatment with medication or fasting glucose level ≥126 mg/dL.

5 Hypercholesterolemia as treatment with medication or a serum cholesterol level ≥240 mg/dL.

6 Hypertriglyceridemia as treatment with medication or a serum triacylglycerol level ≥200 mg/dL.

7 low HDL cholesterol as an HDL cholesterol level <40 mg/dL.

**Table 3.** Common elements of the baseline assessment at both sites

Classification	Contents	Methods
Demographic characteristics	Sex, age, education, marriage, cohabitation, income, subjective economic status, and occupation	Questionnaire/interview
Medical history	Past history of physician-diagnosed diseases (stroke, transient ischemic attacks, myocardial infarction, angina pectoris, heart failure, chronic kidney disease, hypertension, dyslipidemia, diabetes, thyroid disease, fatty liver, chronic hepatitis, liver cirrhosis, asthma or chronic obstructive pulmonary disease, osteoporosis, arthritis, autoimmune disease, and a malignant tumor)	Questionnaire/interview
	Family history of myocardial infarction, hypertension, stroke, and diabetes)	
	Medicine treatment history	
	Reproductive health information (menarche, menopause, pregnancy, gestational diabetes and hypertension, oral contraceptive use, and female hormone use)	
Health-related behaviors	Smoking (lifetime smoking, current smoking, duration, amount, age at initiating smoking)	Questionnaire/interview
	Drinking (lifetime drinking, current drinking, duration, amount, age at initiating drinking)	
	Physical activity (frequency and duration of walking, moderate-intensity, and vigorous activity, using International Physical Activity Questionnaire-Short Form)	
	Sleep and obstructive sleep apnea (bedtime, rise time, sleep duration, obstructive sleep apnea, using Berlin questionnaire)	
	Usual dietary intake (112-item semi-quantitative food frequency questionnaire)	
Psychological health and social support	Depression (Korean version of the Beck Depression Inventory-II)	Questionnaire/self-report
	Stressful life events (Korean version of the life experiences survey questionnaire)	
	Cognitive condition (Korean version of the Mini-Mental State Estimation for dementia screening, only at least 50 years of age)	Questionnaire/interview
	Social network properties	Questionnaire/interview
	Social support from spouse	
Body size and composition	Anthropometric measurements (height, weight, arm circumference, waist circumference, hip circumference, thigh circumference)	Examination
	Bioimpedance (body fat, lean mass, muscle mass, etc.)	
Cardiovascular examination	Single-arm blood pressure: resting blood pressure and pulse	Examination
	Carotid ultrasonography (intima thickness, plaque)	
	Electrocardiogram	
Biochemical indicators	Blood analysis (glucose, insulin, total cholesterol, triglyceride, HDLcholesterol, BUN, creatinine, uric acid, total protein, albumin, AST, ALT, y-GTP, 25-OH vitamin D, hs-CRP, HbAlc, CBC)	Blood, urine
	Urinalysis (proteins, ketones, blood, bilirubin, nitrites)	

HDL, high-density lipoprotein; BUN, blood urea nitrogen; AST, aspartate aminotransferase; ALT, alanine aminotransferase; γ-GTP, gamma-glutamyl transferase, hs-CRP; high-sensitivity C-reactive protein; HbA1c, hemoglobin A1c; CBC, complete blood count.

**Table 4.** Site-specific elements of the baseline assessment

Classification	Contents
Health related behaviors	Physical activity and sleep using a 3-dimensional accelerometer^1^
Body size and composition	QCT^1^
	DXA^2^
Vascular examination	Dual-arm blood pressure^1^
	Central blood pressure, augmentation index^1^
Biochemical indicators	LDL cholesterol^1^
	Hemostatic markers (PT, aPTT, factor VII, factor VIII, fibrinogen, D-dimer)^1^
	Inflammatory markers (IL-1a, IL-p1, IL-6,TNF-a, TNF-p, CD40 ligand)^1^
	Cardiac marker (highly sensitive troponin T)^1^
	Adiponectin^†^, C-peptide^2^
	Heavy metals (lead, cadmium, mercury)^2^
	Persistent organic pollutants (urine arsenic, bisphenol A, etc.)^2^

QCT, quantitative computed tomography; DXA, dual-energy X-ray absorptiometry; LDL, low-density lipoprotein; PT, prothrombin time; aPTT, activated partial thromboplastin time; IL, interleukin; TNF, tumor necrosis factor; YUCM, Yonsei University College of Medicine; AUSM, Ajou University School of Medicine.

1 Only at the YUCM clinic.

2 Only at the AUSM clinic.
